# The approaches and methods of music psychology in the relationship between music emotion and cognition in music teaching activities

**DOI:** 10.3389/fpsyg.2022.1011249

**Published:** 2022-10-04

**Authors:** Nan Jia, Chongze Yang

**Affiliations:** ^1^College of Art, Hebei Normal University of Science and Technology, Qinhuangdao, China; ^2^College of Food Science and Technology, Hebei Normal University of Science and Technology, Qinhuangdao, China

**Keywords:** music teaching, psychology, emotion and cognition, positive emotion, negative emotion

## Abstract

In order to further improve the effect of music teaching, more music psychology should be applied in music teaching to assist teaching, and students should better understand the emotional elements reflected in music through music emotion and cognitive teaching. This essay starts from the relationship between music emotion and cognition, to deeply explore the application of music psychology in teaching activities, through the construction of music education psychological regulation function model to explore the effect of the application of psychology in music teaching. The results showed that the scores of positive emotions were significantly improved, while the scores of negative emotions were significantly decreased. The difference between the improvement and reduction of positive emotions was significant (*p* < 0.01, *p* < 0.01). The results show that psychology based on the relationship between emotions and people is helpful to improve the effectiveness of music teaching. And on this basis put forward the music teaching activity innovation path.

## Introduction

As a special subject, music itself has the deepest power of the people. Music can wash and immerse the heart. Music course is also an important way to implement esthetic education in the process of quality-oriented education, which can better enrich students’ minds, develop students’ phenomenal power, and further enhance students’ phenomenal space and creativity (Au and Lau, 2021). In addition, music can deeply affect students, help students form a correct attitude toward objective facts, enhance students’ moral concepts and moral feelings, and better regulate students’ behavior. The realization of these needs to use the emotional guidance and cognitive concept of music, through the emotional and cognitive guidance of music psychology to better have a profound impact on students’ thoughts, enhance students’ good moral sentiment, increase wisdom and improve health, and promote students to develop good ideological morality (Topal et al., 2021). Music education is not only needed for the construction of socialist spiritual civilization, but also an important means to stimulate students’ musical ability and individualized and comprehensive development. Based on this, from the perspective of music psychology, this essay deeply discusses the application path of the relationship between emotion and cognition in music teaching activities.

## References

Rahiem et al. believe that in the overall activity of music practice, music appreciation is the receiving link of music creation and performance. In the final analysis, the activities of composers and performers, which are for the audience to enjoy, are always centered around the audience. Without music appreciation, music creation and performance will lose their fundamental significance (Rahiem, 2021). An et al. put forward that music appreciation is not only a passive accepting behavior, but also an active and subjective creative activity (An et al., 2022). With the in-depth study of music esthetic practice, modern music esthetics especially turns its attention to the link of music acceptance, and examines the acceptance of music to the same important degree as music creation and performance from a new perspective. Music appreciation is the product of the image activity of the appreciator. Ostendorf et al. pointed out that the emotions expressed or inspired by music are certain, but such certain emotional movement forms may be generated by different people’s attitudes toward different time, so people in emotional movement will seek or recall things that cause similar emotional movement in their own experience. In this way, the definite musical mood also produces the uncertain musical content (Ostendorf et al., 2020). Therefore, when students appreciate the same piece of music, due to their different life experiences, they cannot associate or imagine the music content is exactly the same. Xu et al. believe that the esthetic education function of music is mainly to enrich the emotional experience of esthetic subjects, so as to improve the ability of music appreciation and performance. In the teaching of music appreciation, it is necessary to arouse the enthusiasm of the appreciator, that is, the esthetic subject, so that he can actively, actively and consciously participate in the process of psychological experience. Junior high school students are exposed to a lot of music and have formed certain esthetic standards. Unlike primary school students, they are not easy to accept the esthetic content arranged by teachers (Xu et al., 2021). Moreno, M. et al. pointed out that in music appreciation activities, esthetic subjects always judge esthetic objects with certain esthetic standards. For music works that do not meet their own esthetic standards, they often fail to attract their esthetic attention, resulting in the inability to complete the psychological process of music appreciation (Moreno and Woodruff, 2022). Due to the differences in esthetic personality between junior high school students and teachers, teachers do not pay good attention to the esthetic psychology of teenagers and lack of understanding of the needs of teenagers. As a result, junior high school music appreciation materials are not comprehensive enough, and it is often difficult to arouse the interest of junior high school students in music appreciation class.

## An experimental study of music psychology in regulating students’ psychological function and promoting teaching effect

### Experimental hypothesis and design

*Hypothesis 1*: In terms of music type, there are differences between soundscape music stimulation and non-soundscape music stimulation in the influence of skin electricity, skin temperature, heart rate and EMG of subjects.

*Hypothesis 2*: In terms of music listening methods, abdominal breathing and chest breathing have different effects on skin electricity, skin temperature, heart rate and electromyography.

*Hypothesis 3*: When abdominal breathing is used in music listening, the effect of listening to soundscape music is more significant than that of non-soundscape music in inducing positive emotions.

*Hypothesis 4*: When listening to soundscape music stimuli, abdominal breathing is more effective than chest breathing in inducing positive emotions.

This experiment was a multi-factor completely randomized experimental design (2 × 2 factor experimental design/two-factor experiment), and each subject was treated with four experimental conditions. To avoid the order effect, a 4 × 4 standard Latin square design was adopted (Jannusch et al., 2021). The independent variables of this experiment were two levels of music selection (soundscape music and pure non-soundscape music) and two levels of music listening style (abdominal breathing and chest breathing; see Table 1).

**Table 1 tab1:** Variable selection design table.

	Listening style (B)			
	Soundscape music (a1)	Abdominal breathing (b1)	Thoracic breathing (b2)	
Music choice (A)		O1:b1a1	O2: b2a1	Oa1
	Non-soundscape music(a2)	O3:B1a2	O4: B2a2	Oa2
		Ob1	Ob2	

Respiration is the process of gas exchange between the human body and the outside world, and respiration rate represents the number of individual breaths in a unit of time, the unit is times/min. In this study, “breathing” was determined as an independent variable, and the effects of two levels of breathing, “chest breathing” and “abdominal breathing,” on the physiological indicators of the autonomic nervous system of each subject were investigated (Hashemi et al., 2022). When the emotional state is stressed, the respiratory rate increases. On the contrary, it decreases, and about 70 times/min is the respiratory rate of healthy subjects.

The subjects were college students. A total of 32 subjects, including 12 males and 20 females, aged 18–25 years with an average age of 22.5 years (SD = 1.25 years) were recruited by means of voluntary registration through notices and advertisements. All subjects had no cardiovascular or respiratory diseases, and did not do strenuous exercise 2 h before the test. The scale used in this study is the positive and negative Emotion Scale (Kirk et al., 2022). He revision of PANAS-R scale was based on the theory of affective loop model, and the items of the scale were collected and selected, and a series of experimental tests were carried out. Exploratory factor analysis was used to screen the emotional word items of the scale, and then factor analysis was carried out. The KMO value was 0.781, and the Chi-square value of Bartletts spherical test was 2645.024 (*p* < 0.001). By calculating the CR value, the discrimination degree of each item was tested. The results showed that the CR value of all emotional word items was significant at the level of *p* < 0.001 (see Table 2), indicating that the discrimination degree of items was good.

**Table 2 tab2:** Factor loads, commonality and CR values of PANAS-R items.

Project	Load factorPA	NA	Common degrees	CR value
Active	0.861		0.740	7.602
Enthusiastic	0.859		0.762	13.361
Happy	0.809		0.770	12.752
Elated	0.798		0.669	13.866
Excitedly	0.773		0.599	16.102
Proud	0.763		0.602	12.173
Delighted	0.739		0.565	15.539
Energetic	0.712		0.512	12.827
Grateful	0.567		0.388	14.723
Ashamed		0.750	0.563	8.475
Sad		0.748	0.587	7.386
Afraid		0.745	0.554	10.635
Nervous		0.712	0.509	7.250
Terrified		0.683	0.468	10.420
Guilty		0.572	0.331	8.978
Irritable		0.554	0.335	7.687
Jittery		0.529	0.386	8.283
Irritated		0.461	0.389	6.646

PA, positive emotion; NA, negative emotion; CR value is significant at *P* < 0.001 level. The revised PANAS-R scale included nine words for describing positive emotions and nine words for describing negative emotions, and participants were required to describe the experience of emotional words on a 5-point Likert scale. The internal consistency coefficients were 0.79 and 0.80, respectively.

### The experimental process

#### Preparation: Breathing exercises and pre-test of PANAS-R self-report scale

The behavior laboratory in which this experiment was conducted was quiet and tidy. In the preparation stage of the experiment, indoor temperature and light should be adjusted. Close the blackout curtains and adjust the lighting rheostat to minimize the lighting brightness of the room and create a safe and comfortable music listening atmosphere for the subjects. The indoor temperature is kept at 22°C ± 2°C by air conditioning (Fraenkel, 2020). To avoid interference with music listening and experimental data signals, participants were required to remove necklaces, rings, bracelets, and mobile phones on silent or airplane mode. The subjects sat on the sofa and adjusted to a comfortable posture. The subjects wore the experimental equipment for the subjects. Before the start of the experiment, the subjects read the “Subjects Need to Know,” which included the procedure, abdominal breathing methods and precautions. The experimenter instructed the subjects to perform abdominal breathing exercises.

#### Implementation: Baseline and experimental measurements

The data of this experiment were measured one by one by the subjects, and the experimental program was compiled by E-PRIME2.0 software. The procedure consists of three components: baseline data collection, positive emotion induction and PANAS-R scale filling. The duration of each stage was 127 s, and the scale was filled out after each item of positive emotion was evoked. The experimental conditions for each subject were randomly presented as Latin squares. The specific experimental process is shown in Table 3.

**Table 3 tab3:** Experimental process arrangement.

Conditions	Process							
	127 s	127 s	127 s	127 s	127 s	127 s	127 s	127 s
1	Baseline 1	Soundscape music	Baseline 2	Non-soundscape music	Baseline 3	Soundscape music	Baseline 4	Non-soundscape music
2	Baseline 1	Soundscape music	Baseline 2	Non-soundscape music	Baseline 3	Non-soundscape music	Baseline 4	Soundscape music
3	Baseline 1	Non-soundscape music	Baseline 2	Soundscape music	Baseline 3	Soundscape music	Baseline 4	Non-soundscape music
4	Baseline 1	Non-soundscape music	Baseline 2	Soundscape music	Baseline 3	Non-soundscape music	Baseline 4	Soundscape music

#### Experimental period

In the positive emotion induction stage, the subjects would listen to four musical stimuli in turn, and four beats of the same pitch would appear at the beginning and the end of the music to remind the beginning and the end of the music (Dunbar et al., 2022).

### Results and analysis

#### Self-rating scale report results and analysis

The results of multivariate analysis of variance in Table 4 show that music type and breathing style have significant effects on emotion induction, indicating that corresponding emotions are successfully evoked. The differences between positive emotion and negative emotion induced by different listening methods (abdominal breathing and chest breathing) and different music types (soundscape music and non-soundscape music) were compared, and the difference test was shown in Table 5. Condition I represents soundscape music × abdominal breathing, condition II represents non-soundscape music × abdominal breathing, condition III represents soundscape music × chest breathing, and condition IV represents non-soundscape music × chest breathing.

**Table 4 tab4:** Self-rating scale reports the results of ANOVA.

Emotional type	The mean square	The *F*-value	Sig.
Active	44.681	35.006^***^	0.000
Enthusiastic	38.234	25.392^***^	0.011
Happy	39.011	29.865^**^	0.022
Elated	42.568	40.335^**^	0.031
Excitedly	39.082	22.484^*^	0.041
Proud	31.220	32.609^***^	0.122
Delighted	30.992	26.804^*^	0.023
Energetic	41.221	32.469^***^	0.015
Grateful	30.145	22.557^*^	0.063
Ashamed	0.841	6.358^*^	0.108
Sad	0.216	3.781^*^	0.197
Afraid	1.292	5.880^**^	0.098
Nervous	1.414	4.589^**^	0.235
Terrified	0.291	10.220^*^	0.645
Guilty	1.541	5.667^*^	0.891
Irritable	2.385	3.475^**^	0.100
Jittery	3.013	0.691^*^	0.092
Irritated	2.991	0.407^*^	0.450

**p* < 0.05; ***p* < 0.01; ****p* < 0.001.

**Table 5 tab5:** Difference of positive emotion and negative emotion before and after test under different conditions.

Conditions	Positive emotions (*n* = 32)			Negative emotions (*n* = 32)		
	Pre-test (M ± SD)	Posttest (M ± SD)	Sig.	Pre-test (M ± SD)	Posttest (M ± SD)	Sig.
I	15.89 ± 4.22	23.91 ± 6.14	5.62^***^	14.97 ± 3.49	12.95 ± 2.94	−3.54^**^
II	16.07 ± 5.09	21.64 ± 7.45	4.99^***^	14.33 ± 4.58	13.27 ± 3.96	−3.86^**^
III	16.79 ± 4.22	21.01 ± 6.14	5.62^***^	15.97 ± 3.49	12.95 ± 2.94	−3.54^**^
IV	14.97 ± 5.09	15.02 ± 7.45	4.99^***^	15.33 ± 4.58	15.57 ± 3.96	−3.86^**^

* *p* < 0.05;

** *p* < 0.01;

*** *p* < 0.001.

As can be seen from the above table, in the four experimental conditions of I, II, III, and IV, the scores of positive emotion before and after the test were improved to varying degrees, while the scores of negative emotion before and after the test were decreased to varying degrees, and the difference between the two was significant (*p* < 0.01, *p* < 0.001; Guo and Xiao, 2021). Therefore, the results of the difference test indicate that the manipulation of the four experimental conditions is effective.

In the process of inducing positive emotions, the values of positive emotions before and after the four experimental conditions have been significantly increased. As can be seen from Figure 1, condition I (soundscape music × abdominal breathing) increased the most (pretest =15.89 ± 4.22, posttest =23.91 ± 6.14), followed by condition II (non-soundscape music × abdominal breathing; pretest =16.07 ± 5.09, posttest =13.27 ± 3.96), and condition III again. Soundscape music × chest breathing (pre-test =16.79 ± 4.22, posttest =12.95 ± 2.94), and condition IV, non-soundscape music X chest breathing (pre-test =14.97 ± 5.09, posttest =15.02 ± 7.45) had the smallest increase (Ajmani and Kumar, 2022).

**Figure 1 fig1:** Difference of positive emotion before and after test under different conditions.

In the process of inducing negative emotions, the values of negative emotions before and after the four experimental conditions all decreased significantly and to different degrees. As can be seen from Figure 2, condition III (soundscape music + chest breathing) had the largest reduction (pretest =15.97 ± 3.49, posttest =21.01 ± 6.14), and condition I (soundscape music + abdominal breathing) had the second largest reduction (pretest =14.97 ± 3.49, posttest =12.95 ± 2.94). Condition II, non-soundscape music + abdominal breathing (pretest =14.33 ± 4.58, posttest =21.64 ± 7.45), and condition IV, non-soundscape music + chest breathing (pretest =15.33 ± 4.58, posttest =15.57 ± 3.96) had the smallest reduction (Garg et al., 2022).

**Figure 2 fig2:** The difference of negative emotions measured before and after different conditions.

#### Test and analysis of significant differences in physiological indicators

Table 6 shows the descriptive statistical results of skin temperature (STS), galvanic skin (SCR), heart rate (BVP) and electromyography (EMG) of the dependent variables of this study, including mean (M) and standard deviation (SD).

**Table 6 tab6:** Descriptive statistical results of physiological indicators.

	Soundscape music (*n* = 32)				Non-soundscape music (*n* = 32)			
	Abdominal breathing		Thoracic breathing		Abdominal breathing		Thoracic breathing	
	M	SD	M	SD	M	SD	M	SD
STS	1.9531	1.2468	1.66647	0.9332	0.113888	1.71809	−0.009783	0.75689
SCR	−7.02722	2.061785	−5.014174	2.0639674	−3.396138	2.0639679	−1.574833	1.529027
BVP	−8.056602	1.3467893	−3.772575	1.4263564	−2.58998	1.5641307	−0.0737	1.093805
EMG	−10.22204	3.0723889	−4.759364	3.6875054	−4.879805	2.2548016	0.580964	2.5944441

##### Skin temperature (STS) index difference test analysis

According to the results of ANOVA (Table 7), in terms of STS index, there was a significant difference in music condition between the two experimental conditions (*p* < 0.005^***^), while there was no significant difference in breath between the two experimental conditions (*p* > 0.05). There was no significant interaction between music type and breathing mode (*p* > 0.05; Guimares, 2021).

**Table 7 tab7:** Results of within-subject effect test of skin temperature (STS) index.

The source	Type III sum of squares	df	The mean square	F	Sig.	Partial Eta square
Music	98.868	1	98.868	75.667	0.000	0.709
Error (music)	40.501	31	1.300			
breath	1.344	1	1.346	0.723	0.402	0.024
Error (breath)	57.653	31	1.860			
Music * breath	0.214	1	0.211	0.204	0.655	0.007
Error (music * breath)	32.412	31	1.045			

##### The difference test and analysis of electric skin (SCR) index

According to Table 8, in terms of SCR index, the intervention effect of soundscape music was better than that of non-soundscape music under the two conditions (*p* < 0.005^***^). There were significant differences between abdominal breathing and thoracic breathing under the two music conditions (*p* < 0.001^***^), but no significant interaction (*p* > 0.05).

**Table 8 tab8:** Results of intra subject effect test of electroskin (SCR) index.

Test for intra-subject contrast in SCR						
The source	Type III sum of squares	df	The mean square	F	Sig.	Partial Eta square
Music	399.931	1	399.935	77.941	0	0.714
Error (music)	159.054	31	5.132			
Breath	117.627	1	117.622	21.571	0	0.410
Error (breath)	169.045	31	5.453			
Music * breath	0.293	1	0.294	0.095	0.758	0.003
Error (music * breath)	95.232	31	3.075			

##### Heart rate (BVP) index difference test analysis

According to the descriptive statistical results (Tables 9, 10), there was a significant difference between the two experimental conditions of music type and breathing mode (*p* < 0.005^***^), and the main effect was significant (*p* < 0.005^***^) in BVP index (Raj et al., 2021). Further paired sample *t*-test showed that there was a significant difference between chest breathing and abdominal breathing under soundscape music condition (*p* < 0.005^***^). The difference between chest breathing and abdominal breathing was significant (*p* < 0.005^***^) under the condition of non-soundscape music. In chest breathing condition, there was a significant difference between soundscape music and non-soundscape music (*p* < 0.005^***^). In abdominal breathing condition, the difference between soundscape music and non-soundscape music was significant (*p* < 0.005^***^).

**Table 9 tab9:** Results of within-subject effect test of heart rate (BVP) index.

Test for intra-subject contrast of BVP					
The source	Type III sum of squares	df	The mean square	F	sig.
Music	672.063	1	672.068	450.21	0.000
Error (music)	46.271	31	1.492		
Breath	369.946	1	369.945	214.20	0.000
Error (breath)	53.541	31	1.727		
Music * breath	25.001	1	25.002	11.023	0.002
Error (music * breath)	70.296	31	2.268		

**Table 10 tab10:** Test results of paired samples of heart rate (BVP) index.

Paired sample *T*-test		M	sD	Standard error of the mean	95% confidence interval		t	df	Sig.
					The lower limit	Upper limit			
1	SM AB vs. TB	−4.2840353	2.1212586	3,749,892	−5.0488304	−3.5192398	−11.425	31	0
2	NSM AB vs. TB	−2.5162085	1.8680951	3,302,358	−3.1897285	−1.8426887	−7.619	31	0
3	AB SM vs. NSM	−5.4666992	1.9948600	3,526,430	−6.1859191	−4.7474792	−15.502	31	0
4	TB SM vs. NSM	−3.6988725	1.8817799	3,326,549	−4.3773263	−3.0204184	−11.119	31	0

According to the descriptive statistical results of EMG indexes (Table 11), there was a significant difference between the two intervention conditions of soundscape music and non-soundscape music in EMG index (*p* < 0.000^***^), but no significant interaction (*p* > 0.05). The intervention effect of SM was better than that of NSM in AB and TB respiratory conditions (*p* < 0.000^***^). In SM and NSM, there was a significant difference between abdominal breathing and chest breathing (*p* < 0.000^***^), and the effect of abdominal breathing was better than that of chest breathing (*p* < 0.000^***^).

**Table 11 tab11:** Results of intra-subject effect test of electromyography (EMG) index.

Test for intra-subject contrast of BVP					
The source	III type of sum of squares	df	The mean square	F	Sig.
Music	912.932	1	912.931	94.566	0.000^***^
Error (music)	299.275	31	9.653		
Breath	954.571	1	954.58	109.830	0.000^***^
Error (breath)	269.438	31	8.692		
Music * breath	2.87E-05	1	2.87E-05	0.000	0.998
Error (music * breath)	181.984	31	5.871		

## The path and method of music psychology in music teaching

### Improve the teaching effect by regulating function model of music psychological education

The music education resource model (Figure 3) is built on the basis of students’ age development and ability level. The content reflects the potential scope and target of music education inside and outside the school, that is, all the resources that music education can provide for students. The latent function model of music education (Figure 4) shows the influence of primary music education on individual students and the relationship among various dimensions (Chaturvedi et al., 2021).

**Figure 3 fig3:** Hargreaves’ model of music education resources.

**Figure 4 fig4:** Hargreaves’ potential functional model of music education.

The music education resource model is built on three polar dimensions. First, the vertical dimension of the model represents a series of formal resources for the institutionalized training of music education and a variety of other informal resources; Secondly, the horizontal dimension separates the resources inside and outside the school of music education. The resources inside the school represent the prescribed resources provided by the school, while the resources outside the school represent the resources that students can choose independently. Third, in the “professional-general” dimension, it includes professional resources and general resources in music education (Das and Satpathy, 2021).

The realization of the music education psychological adjustment function model (see Figure 5) includes two dimensions: measurement method and influencing factors. The measurement methods of music-induced emotions include self-report scale measurement, physiological index measurement and behavioral intervention measurement. The measurement results are reflected in the three influencing factors of music-induced emotions, which are individual factors, music ontological characteristics and breathing mode characteristics.

**Figure 5 fig5:** Psychological adjustment function model of music education.

### Strengthen the understanding and cognition of music works appreciation practice

#### Inspire the initiative of students’ esthetic thinking

Some teachers in the music appreciation class always in a commanding attitude, stiff and rigid to teach students what the music is the background of The Times, what is the expression of thoughts and feelings, how to understand the music and so on. Such rational analysis and blunt loss is often very easy to make students lose interest, resulting in the generation of students disgust and weariness. Therefore, in the process of teaching, the teacher and the educatees should and are allowed to have certain differences in the emotional understanding of music works, which is the law of human understanding of objective things. If you insist on consistency, it is tantamount to swallowing dates in a circle and mass production (Huang and Yang, 2022). Therefore, students should be appropriately encouraged to show their individuality, encourage students to expand their imagination with music, enter the rich emotional atmosphere of music works, and enhance the inside information. In music education, it is of special significance to pay attention to the development of students’ personality. Music is an experiential subject, only the active participation and independent experience of students can feel the happiness of learning and accumulate learning results. In the teaching of music appreciation, teachers guide students to participate actively, give full play to their main role, mobilize the enthusiasm and initiative of students’ active participation in learning, so that students can really get audio-visual, singing, thinking ability and imagination exercise in music appreciation, and deepen their own music perception and esthetic power in emotional experience. In addition, because of the strong practicality of music art, it is closely related to other forms of practical activities. In appreciation class, attention should be paid to students’ participation and practice, to students’ feelings, experience, understanding and expression of music emotion, and to students’ feelings, experience, performance and appreciation of music beauty, so that students can understand music through profound experience rather than preaching (Davies et al., 2021). We should appreciate the teaching, understand the expressive force of music works, experience the rich spiritual feelings that music brings us, cultivate students to understand the ability of human beings to understand the world with music mode. The teaching effect of music appreciation is directly related to the effect of music education and whether our education can achieve those positive social effects we want.

#### Protect the freedom of students’ esthetic imagination

It is normal for people to have different understandings of music. It is the non-semantic nature and uncertainty of music that provide a wide space for people’s different imagination and association, laying the foundation for creative musical thinking activities. Many people, including music teachers, agree that music education should cultivate students’ imagination in theory, but there is often no space for students’ imagination to play in concrete teaching practice. There are many reasons for this situation, but the fundamental reason is that students cannot be treated correctly, treated as learning subjects and given equal status in music learning (Bakerjian et al., 2020). As a matter of fact, due to the open growing environment and diversified ways of receiving education, today’s students may understand all kinds of new things and new knowledge more quickly and widely than adults, so that they have more information mastery and understanding of new things than adults. They have no inherent views, and there is often no framework for music learning and understanding, and no discipline rules and regulations. However, with the advantages of sensitivity to new culture, recognition and acceptance ability, they show a natural nature and vitality of learning. Some students said their feelings about music learning like this, “I think the school music class is boring, I feel like learning. There are steps, there is analysis, there is what there is a formula for what this music is like, right (Zhao et al., 2019). Why is it not what I think, and why is it wrong? “Some students think that” for music, I think I only need my own feeling, which is not clear, and maybe it will bump into the feeling in my heart inadvertently. To achieve this feeling, I cannot restrict my “freedom,” freedom from external interference. If everyone had to understand music by “rules,” then “music would not have a feel.” It can be seen that students’ “rebellion” against music education in the traditional sense is not a whim, but a positive thinking based on independent learning, full of critical spirit, and there is no lack of insight.

### Cultivate students’ music esthetic ability by creating teaching situation

#### Create situations with instrumental props to stimulate students’ interest

In the music class, the use of small and convenient instruments to assist teaching is conducive to students’ immersive experience of music. The necessary piano in the traditional music classroom can no longer satisfy students’ curiosity about the timbre of various Musical Instruments. The use of small instruments in teaching can stimulate students’ interest in learning. When using small instruments, students can easily immerse themselves in the real music situation and feel the charm of Musical Instruments (Ebrahimi et al., 2022). The sound of some small instruments is clear and pleasant, and it is easy to express the happy mood of music works. At the beginning of the class, students are first exposed to the small instruments that can express the emotion of the works, so that they can experience the emotional content of the textbook in advance by using the situation created by physical instruments, and further enhance their esthetic experience.

#### Use things around you to create a situation, stimulate learning enthusiasm

Music comes from life, and students’ life is full of music. When teaching, if students can choose music that is familiar with and related to teaching content as an intermediary, they will get twice the result with half the effort. When introducing the content, we should also pay attention to the methods and methods, and when selecting the content, we should try our best to select the content that students feel close to, so as to create a teaching situation close to the content of the work and students’ preferences, and stimulate strong enthusiasm for learning.

#### Teaching stories creates situations and arouses students’ interest

An interesting story is easy to arouse students’ interest. When preparing lessons, the author will create story situations related to the content of music textbooks in advance to make students intoxicated as much as possible, and then transfer their interest to the music works to be learned. The story should not be long, but it should be relevant to the book.

#### Set up questions to arouse students’ enthusiasm

Junior high school students have the psychological characteristics of curiosity and competitive, teachers can use this psychological characteristics to set up suspense, guessing links. When teaching, the author also asks students to listen to music segments and release pictures of Musical Instruments to ask what kind of Musical Instruments are played (Sharma and Kumar, 2019). This fully mobilized the competitive heart of students, and they have been scrambling to answer, actively participate in the music esthetic activities. Students also gain a better understanding of the timbre of different Musical Instruments, laying a solid foundation for future music study.

#### Set up game links to create situations and activate the teaching atmosphere

Setting up interesting games in music teaching can greatly ignite students’ interest in learning. In the teaching practice, the author also set up a lyric filling game combined with the teaching content. These interesting games greatly stimulated the enthusiasm of students to learn this course.

### Explore the musical emotional elements in music works

#### Analysis of music elements

Music classroom takes music esthetic education as the core, and teachers’ teaching goal is to improve students’ esthetic appreciation level as the main goal. Only by letting students understand the specific content of many musical elements of music and how different forms of expression of the elements reflect the emotion of the work can they experience the beauty of music to the greatest extent. The movement form of music is similar to the movement state of human psychology, so music can express people’s mental state and emotional thoughts in an abstract way. In order to cultivate students’ esthetic ability by listening to and appreciating music, it is not enough to allow them to listen to and appreciate the psychological fluctuations. It is necessary to guide them to master the internal association between music sound and its object of expression, and understand how the specific operation of music expression affects the changes in the emotional content of the object of expression. Therefore, only staying in the physiological perception cannot meet the students’ esthetic needs for music. It is necessary to conduct systematic study to master the basic elements of music and the importance of music elements to the expression of content. The enhancement of students’ music esthetic experience and the cultivation of esthetic ability need to start with the basic elements of music ontology in works.

#### Understand the cultural background

Music belongs to the category of human culture. While teaching music knowledge and skills in music classroom, the cultural and historical background related to music should not be underestimated. Teachers need to expand the cultural connotation as much as possible, so that students can actively obtain the cultural content contained in the works in the process of music esthetics, further cultivate artistic sentiment, and improve the overall quality (Hekmati et al., 2021). Understanding the historical background of music works is to enhance the horizontal connection between music lessons and other disciplines. It is the main way to improve the esthetic understanding of music. It can help students deepen their perception of music through the understanding of history and culture, and understand the characteristics of music styles in different times. This is the most common way to teach a musical composition and the life of a musician. Through the teacher’s teaching, students can accept the historical background, humanistic influence and the composer’s life experience when the work was created. It is easy for students to understand the mood of the composer when he created the work, which is helpful for students to understand and analyze the emotion of the work.

## Conclusion

This research focuses on the realization of the psychological regulation function of music education, which is the core issue, and takes music education activities to induce positive emotions as the realization approach. The selection and design of research methods strictly follow the norms of mixed method research. First of all, the main conclusions of this study are summarized as a whole: this study defines relevant concepts on the basis of searching, sorting, analyzing and commenting on “music education function research” and “music evoked emotion research.” Then mixed methods are used to carry out the main research, among which the experimental research on the psychological regulation function of music education belongs to the quantitative research stage of mixed methods, and the qualitative intervention research on the psychological regulation function of music education belongs to the qualitative research stage. The analysis of the factors influencing the realization of the psychological adjustment function of music education based on the two methods is an integrative study in the mixed method. The hybrid method provides the methodological support for the main part of the whole research, and also provides the theoretical basis for the research findings. The research findings include the model construction of the psychological regulation function of music education and the prospect of the educational value of this model. The mechanism of music education activities to induce positive emotions is the sublimation of the theoretical basis of music education psychological regulation function. Based on the literature review of “music education function” and “music evoked emotion,” the mechanism of music education activities to induce positive emotion originates from the further interpretation of the mechanism of music evoked emotion. Specifically, music education activities induce positive emotion mechanism is mainly manifested in the relationship between music and emotion of four models (in theory), including music clues consistency model, music expectation model, music emotion of synergy theory and multiple mechanism model, in which multiple mechanism model, including seven kinds of independent existence mechanism, they are brainstem reflex, rhythmic synchronization, evaluative reflex, emotional infection, visual imagination, episodic memory and musical anticipation.

## Data availability statement

The original contributions presented in the study are included in the article/supplementary material, further inquiries can be directed to the corresponding author.

## Author contributions

NJ contributed to the writing of the manuscript and data analysis. CY supervised the work and designed the study. All authors contributed to the article and approved the submitted version.

## Conflict of interest

The authors declare that the research was conducted in the absence of any commercial or financial relationships that could be construed as a potential conflict of interest.

## Publisher’s note

All claims expressed in this article are solely those of the authors and do not necessarily represent those of their affiliated organizations, or those of the publisher, the editors and the reviewers. Any product that may be evaluated in this article, or claim that may be made by its manufacturer, is not guaranteed or endorsed by the publisher.

## References

[ref1] AjmaniN.KumarS. (2022). The struggles of self: analysing the music of linkin park and sleeping at last. Hum. Arenas 5, 161–178. doi: 10.1007/s42087-020-00129-3

[ref2] AnH.SungW.YoonS. Y. (2022). Hands-on, minds-on, hearts-on, social-on: a collaborative maker project integrating arts in a synchronous online environment for teachers. TechTrends 66, 590–606. doi: 10.1007/s11528-022-00740-x, PMID: 35531261PMC9060412

[ref3] AuT. C.LauN. S. (2021). Private music teachers' knowledge of and attitudes toward students with autism spectrum disorder. J. Autism Dev. Disord. 51, 4551–4559. doi: 10.1007/s10803-020-04809-533559017

[ref4] BakerjianA. D.KbA.AmcA.LaA.StB. (2020). The impact of music and memory on resident level outcomes in California nursing homes. J. Am. Med. Dir. Assoc. 21, 1045–1050.e2. doi: 10.1016/j.jamda.2020.01.103, PMID: 32146039PMC8121202

[ref5] ChaturvediV.KaurA. B.VarshneyV.GargA.KumarM. (2021). Music mood and human emotion recognition based on physiological signals: a systematic review. Multimedia Syst. 28, 1–24. doi: 10.1007/s00530-021-00786-6

[ref6] DasS.SatpathyS. (2021). Multimodal music mood classification framework for kokborok music. Solid State Technol. 63, 5320–5331. doi: 10.1007/978-981-33-4299-6_14

[ref7] DaviesC.ShurdingtonJ.MurrayK.SlaterL.PearsonD. (2021). Music for wellness in rehabilitation patients: programme description and evaluation results. Public Health 194, 109–115. doi: 10.1016/j.puhe.2021.02.008, PMID: 33878712

[ref8] DunbarR.PearceE.TarrB.MakdaniA.BamfordJ.SmithS.. (2022). Author correction: cochlear sgn neurons elevate pain thresholds in response to music. Sci. Rep. 12:1. doi: 10.1038/s41598-022-04978-635017651PMC8752849

[ref9] EbrahimiH.HosseinzadehM.SarayR. S.WilsonM.AreshtanabH. N. (2022). Ability of older adults to recognize cognitive changes and its relationship with mental health: a cross-sectional study. BMC Geriatr. 22, 1–7. doi: 10.1186/s12877-022-03096-235525932PMC9077964

[ref10] FraenkelP. (2020). Integrating music into couple therapy theory and practice. Clin. Soc. Work. J. 48, 319–333. doi: 10.1007/s10615-020-00755-y

[ref11] GargA.ChaturvediV.KaurA. B.VarshneyV.ParasharA. (2022). Machine learning model for mapping of music mood and human emotion based on physiological signals. Multimed. Tools Appl. 81, 5137–5177. doi: 10.1007/s11042-021-11650-0

[ref12] GuimaresJ. P. (2021). Beyond the pulp vanguard: Bruce andrews's film noir series and the dead-end of escapist experimentalism. CounterText 7, 467–500. doi: 10.3366/count.2021.0247

[ref13] GuoZ.XiaoZ. (2021). Research on online calibration of lidar and camera for intelligent connected vehicles based on depth-edge matching. Nonlinear Eng. 10, 469–476. doi: 10.1515/nleng-2021-0038

[ref14] HashemiY.ZaraniF.HeidariM.BorhaniK. (2022). Purposes of internet use among iranian university students: exploring its relationship with social networking site (sns) addiction. BMC Psychol. 10, 1–9. doi: 10.1186/s40359-022-00745-435351206PMC8966315

[ref15] HekmatiI.RanjbarH. A.EskinM.DrakeC. E.JobsonL. (2021). The moderating role of experiential avoidance on the relationship between cognitive fusion and psychological distress among iranian students. Curr. Psychol. 1–8. doi: 10.1007/s12144-021-01539-4

[ref16] HuangR.YangX. (2022). Analysis and research hotspots of ceramic materials in textile application. J. Ceram. Process. Res. 23, 312–319. doi: 10.36410/jcpr.2022.23.3.312

[ref17] JannuschT.ShannonD.VoellerM.MurphyF.MullinsM. (2021). Smartphone use while driving: an investigation of young novice driver (ynd) behaviour. Transport. Res Part F Traffic Psychol. Behav. 77, 209–220. doi: 10.1016/j.trf.2020.12.013

[ref18] KirkU.NgnoumenC.ClauselA.PurvisC. K. (2022). Effects of three genres of focusmusic on heart rate variability and sustained attention. J. Cogn. Enhance. 6, 143–158. doi: 10.1007/s41465-021-00226-3

[ref19] MorenoM.WoodruffE. (2022). Synthesizing advancements in methodology and technology to understand affective expression and music stimuli: a literature review. SN Soc. Sci. 2, 1–18. doi: 10.1007/s43545-022-00335-634934956

[ref20] OstendorfA. L.SchlüterH.HacklnderR. (2020). Sounds in the classroom: auditory context-dependent memory in school-aged children. Open Psychol. 2, 106–118. doi: 10.1515/psych-2020-0101

[ref21] RahiemM. (2021). Storytelling in early childhood education: time to go digital. Int. J. Child Care Educ. Policy 15, 1–20. doi: 10.1186/s40723-021-00081-x

[ref22] RajM.ManimegalaiP.AjayP.AmoseJ. (2021). Lipid data acquisition for devices treatment of coronary diseases health stuff on the internet of medical things. J. Phys. Conf. Ser. 1937:012038. doi: 10.1088/1742-6596/1937/1/012038

[ref23] SharmaA.KumarR. (2019). Risk-energy aware service level agreement assessment for computing quickest path in computer networks. Int. J. Reliab. Saf. 13:96. doi: 10.1504/IJRS.2019.097019

[ref24] TopalA. D.GeerA. K.BudakE. O. (2021). An analysis of the utility of digital materials for high school students with intellectual disability and their effects on academic success Universal Access in the Information Society, 1–16.10.1007/s10209-021-00840-0PMC844264634539303

[ref25] XuL.ZhengY.XuD.XuL. (2021). Predicting the preference for sad music: the role of gender, personality, and audio features. IEEE Access 9, 92952–92963. doi: 10.1109/ACCESS.2021.3090940

[ref26] ZhaoX. L.LiuX.LiuJ.ChenJ.FuS.ZhongF. (2019). The effect of ionization energy and hydrogen weight fraction on the non-thermal plasma vocs removal efficiency. Journal of physics D. Appl. Phys. 52:145201. doi: 10.1088/1361-6463/aafe8b

